This article has been retracted.

# Nomogram Prediction Model Analysis of Risk Factors for Conversion to Thoracotomy after Thoracoscopic Resection of Lung Cancer and Prognostic Value of Lung Cancer

**DOI:** 10.1155/2022/3628335

**Published:** 2022-07-25

**Authors:** Peng Su, Yonggang Zhu, Huilai Lv, Jian Zhang, Chao Huang, Fan Zhang, Ziqiang Tian

**Affiliations:** Department of Thoracic Fifth, Fourth Hospital of Hebei Medical University, Shijiazhuang, 050011 Hebei, China

## Abstract

This study was aimed at exploring the risk factors for thoracotomy in patients undergoing thoracoscopic resection of lung cancer and further analyzing the factors affecting the prognosis of patients. Ninety-six patients with non-small-cell lung cancer who underwent thoracoscopic pulmonary resection were recruited as the subjects, and they were enrolled into the thoracoscopic group (*n* = 88) and the thoracotomy group (*n* = 8) according to whether thoracotomy was performed. Univariate analysis and logistic multivariate regression were performed to analyze the risk factors for conversion to thoracotomy, and nomogram prediction model was employed to analyze the prognostic factors. The results revealed that the proportion of patients over 65 years old, with history of coronary heart disease, diabetes, and pulmonary tuberculosis, etc., in the thoracotomy group and the thoracoscopic group was significantly different (*P* < 0.05). There were statistically significant differences in the development of interlobular cleft, pleural adhesion, tumor diameter > 3.5 cm, vascular and lymph node invasion, and tumor TNM stage between the thoracotomy group and the thoracoscopic group (*P* < 0.05). Overall, the age of patients ≥ 65 years old, tumor diameter > 3.5 cm, hypoplasia of interlobular fissure, history of pulmonary tuberculosis, pleural adhesion, and TNM stage IIIa were all independent risk factors for thoracoscopic resection of lung cancer to thoracotomy. Cox model and nomogram prediction model analysis showed that surgery methods, tumor diameter > 3.5 cm, chemotherapy cycle < 4, chemotherapy, and TNM stage IIIa were all independent factors influencing the prognosis of patients undergoing thoracoscopic lung cancer resection. This nomogram prediction model had high application value in patient prognosis prediction.

## 1. Introduction

Lung cancer is a malignant tumor that mainly originates from the mucosal epithelium of the bronchus and is classified into small-cell carcinoma and non-small-cell carcinoma according to the histological lesions [1]. Non-small-cell lung cancer includes squamous cell carcinoma and adenocarcinoma. Compared with small-cell carcinoma, large-cell carcinoma has slower leukocyte growth and division and relatively late diffusion and metastasis. Non-small-cell lung cancer accounts for about 80% of lung cancers, and most patients are already in the middle and advanced stage when they are discovered, with low 5-year survival [2, 3]. In recent years, with the serious air pollution and the gradual deterioration of the environment, the incidence of various lung diseases is on the rise, among which lung cancer has become one of the cancers with the highest incidence [4]. Data from the National Cancer Center showed that in 2020, the number of new lung cancer cases in China will reach 816,000, accounting for 17.9% of all cancers [5]. That is an average of 16 people getting sick every 10 minutes. 719,000 cases died, accounting for 23.8% of all cancers [6, 7]. Related studies found that the occurrence of lung cancer is mainly caused by the comprehensive effect of in vivo and in vitro factors in patients. In addition, it is also correlated with smoking or smoking history, harmful substances in the environment, family history of diseases, lung or respiratory diseases, and dietary habits [8, 9]. Clinical diagnosis depends on pathological examination. In addition, chest CT, positron emission computed tomography (PET-CT), magnetic resonance imaging (MRI), and other methods can be used for early diagnosis of lung cancer to help doctors understand tumor metastasis and stage the tumor [10, 11].

The type and stage of lung cancer to formulate corresponding treatment measures are necessary to evaluate, such as surgical resection, radiotherapy, or concurrent radiochemotherapy. For patients with advanced lung cancer or patients prone to remote metastasis, radiotherapy, immunotherapy, or a combination of multiple methods may be required [12, 13]. Early lung cancer can be eradicated by surgical resection of tumor tissue and its surrounding tissues. However, common thoracotomy will cause great trauma to patients and require a long time to recover [14, 15]. Video-assisted thoracoscopic surgery was introduced into thoracic surgery in the last century. It has gradually matured and has been widely used in the treatment of benign and malignant thoracic diseases. Avery et al. [16] found that thoracoscopic surgery had the advantages of smaller incision and faster recovery compared to traditional thoracotomy. In a minimally invasive way, the thoracoscopic tube is probed into the lung of the patient to explore and remove the tumor, resulting in small wounds for the patient, thus accelerating the recovery speed of the patient, improving the recovery effect, alleviating the pain of the patient, and preventing and avoiding postoperative infection and complications to a certain extent [17, 18]. However, Jiao et al. [19] found that due to the relatively difficult thoracoscopic surgery, special circumstances such as bleeding and unclear separation of hilar structure during the operation may lead to thoracotomy, and the probability of thoracotomy is still high.

Although there are many studies on the risk factors and prognostic analysis of patients undergoing thoracotomy after lung cancer resection, there is still a lack of reliable and universal statistical prediction methods, so in-depth research is needed. Nomogram is believed to be an evidence-based and accurate prognostic evaluation method, which has been widely used in a variety of malignant tumors. Therefore, nomogram prediction model was employed to analyze the risk factors for thoracotomy in patients undergoing thoracotomy, and the factors influencing the prognosis of patients were analyzed, so as to provide some basis for the treatment of lung cancer.

## 2. Materials and Methods

### 2.1. Research Objects

In this study, 96 patients with non-small-cell lung cancer who underwent thoracoscopic pulmonary resection in our hospital from May 2016 to May 2018 were recruited. Of which, 46 were male patients and 50 were female patients, aged 20-78 years. This study had been approved by the ethics committee of the hospital, and patients and their families had understood the research content and methods and had agreed to sign the corresponding informed consent forms.

Inclusion criteria were as follows: (i) all patients met the diagnosis and treatment guidelines of NSCLC and were confirmed by pathological examination; (ii) no radiotherapy or chemotherapy was given two months before study participation; (iii) no severe acute or chronic infection and other diseases affecting blood routine results; (iv) no distant head and abdominal metastasis and no mediastinal lymph node enlargement or pleural hypertrophy; and (v) patients with normal coagulation function and platelets.

Exclusion criteria were as follows: (i) patients with incomplete clinical data and history information (tumor size, clinicopathological stage (TNM), etc.); (ii) patients with mental illness and unable to cooperate with research; (iii) patients with obvious pleural calcification in active stage of pulmonary tuberculosis; (iv) patients with serious insufficiency of heart function and liver and kidney function; (v) patients with autoimmune diseases; and (vi) patients accompanied by obvious lymphadenopathy.

### 2.2. Patient Data

Age (<65 years old or ≥65 years old), gender (male or female), smoking history (with or without), history of coronary heart disease (with or without), history of tuberculosis (yes, no), history of diabetes (with or without), and other general information were collected. Surgical time, surgical method (simple lobectomy, combined lobectomy, and segmental resection of the lung), and other surgical conditions were recorded. TNM stages (I, IIa, IIb, and IIIa), degree of differentiation (low differentiation, medium differentiation, and high differentiation), histological morphology (squamous cell carcinoma, adenocarcinoma, and large-cell carcinoma), vascular invasion (with or without), lymph node invasion (with or without), and tumor location (right lung or left lung) were collected. Tumor diameter (>3.5 cm or ≤3.5cm) and other pathological conditions were recorded. Postoperative chemotherapy (with or without), pleural adhesion (with or without), interlobular fissure development (complete or incomplete), and other conditions were recorded. The changes of clinical case data of NSCLC patients were observed.

### 2.3. Surgical Treatment and Postoperative Follow-Up

All patients were treated with single-port thoracoscopic surgery. Preoperative blood routine examination, urine routine examination, biochemical indicators, etc., were inspected. After general anesthesia, the patients were placed in lateral supine position, and the healthy side of the lung was ventilated with one lung. The order of thoracoscopic operation was basically the same as that of traditional thoracotomy, the surgical method for carcinoma in situ or noninvasive adenocarcinoma of lung was segmentectomy and lymph node sampling, and the surgical method for other primary lung cancer was lobectomy and systematic lymph node dissection.

The patients were followed up once every 3 months after 12 months, once every 6 months from 24 to 36 months, and once a year after that. Follow-up included chest CT, routine physical examination, and hematology examination. Postoperative recurrence was observed. Recurrence was considered as new lesions at surgical margin, ipsilateral or contralateral hemithorax, mediastinum, etc.

### 2.4. COX Proportional Risk Regression Model

The basic form of COX proportional risk regression model is shown in

(1) $$\begin{array}{c} h\left(t\right)=h_{0}\left(t\right)\exp\left(\beta_{1}x_{1}+\beta_{2}x_{2}+\cdots +\beta_{p}x_{p}\right). \end{array}$$

*x*_1_, *x*_2_,…, and *x*_*p*_ are the independent variables. *β*_1_, *β*_2_,…, and *β*_*p*_ are the partial regression coefficients of independent variables. *h*_0_(*t*) is the risk function at time *t* when *x*_1_ = *x*_2_ = ⋯*x*_*p*_ = 0, which is called the baseline risk function. *h*(*t*) is the risk function of the individual with independent variable *x*_1_, *x*_2_,…, and *x*_*p*_ at time *t*. COX models make no assumptions about the content of the first factor *h*_0_(*t*), while the second factor has parametric models. All COX models are semiparametric models. COX model has two basic assumptions as follows.

- Equal proportion risk assumption: the effect of research factors has nothing to do with *h*_0_(*t*) and time and does not change with the change of time. This assumption is a prerequisite for the establishment of COX regression models (data analysis is of great concern and is generally tested). The effect of research factors is usually expressed in the hazard ratio (HR) as

(2) $$\begin{array}{c} \text{HR}=\frac{h_{i}\left(t\right)}{h_{j}\left(t\right)}=\frac{h_{0}\left(t\right)\exp\left(\beta_{1}x_{i1}+\beta_{2}x_{i2}+\cdots +\beta_{p}x_{ip}\right)}{h_{0}\left(t\right)\exp\left(\beta_{1}x_{j1}+\beta_{2}x_{j2}+\cdots +\beta_{p}x_{jp}\right)} \end{array}$$

(II) Log-linear assumption: the logarithmic risk ratio should have a linear relationship with the independent variables in the model, namely,

(3) $$\begin{array}{c} \text{In}\left[\frac{h\left(t\right)}{h_{0}\left(t\right)}\right]=\text{InHR}=\beta_{1}x_{1}+\beta_{2}x_{2}+\cdots +\beta_{p}x_{p} \end{array}$$

The Kaplan-Meier curves and logrank tests are single-factor analyses that study the relationship between a single variable and survival, and the single-factor analysis is only applicable to categorical variables, not numerical variables, such as gene expression in malignant tumors [20]. In the single-factor survival analysis, the survival function (or cumulative survival rate) is *S*(*t*, *x*), where *S* represents the probability that the survival time of the research object *T* is greater than a specific moment *t*, *x* represents the independent variable (a processing factor), and its assignment rule is shown in

(4) $$\begin{array}{c} x=\left\{\begin{array}{c} 0,\text{No treatment factor},\\ 1,\text{Treatment factors}. \end{array}\right. \end{array}$$

The risk of patients in a treatment group at time *t* is shown in

(5) $$\begin{array}{c} W\left(t\right)=w_{0}\left(t\right)\times \exp\left(\beta \right). \end{array}$$

The risk of the control group at time *t* is shown in

(6) $$\begin{array}{c} W\left(t\right)=w_{0}\left(t\right), \end{array}$$

(7) $$\begin{array}{c} \text{Relative risk degree}=\frac{\text{Handling group risks}}{\text{Control group risk}}=\frac{w_{0}\left(t\right)\times \exp\left(\beta \right)}{w_{0}\left(t\right)}=\exp\left(\beta \right). \end{array}$$

The death function is as follows:

(8) $$\begin{array}{c} D\left(t,x\right)=1-S\left(t,x\right), \end{array}$$

where *D* represents the cumulative mortality rate observed and followed up to time *t*. The death density function is the derivative of

(9) $$\begin{array}{c} m\left(t,x\right)=D\left(t,x\right), \end{array}$$

where *m* represents the death density function (i.e., the instantaneous death rate at time *t*). The risk function is

(10) $$\begin{array}{c} w\left(t,x\right)=\frac{m\left(t,x\right)}{S\left(t,x\right)}, \end{array}$$

where *w* is the risk function, which represents the ratio of instantaneous mortality at time *t* to the number of survivors at time *t* (conditional instantaneous mortality).

### 2.5. Statistical Methods

SPSS 23.0 software package was used for statistical analysis in this study. The Shapiro-Wilk test was used to verify whether the data were normally distributed. The measurement data in accordance with the normal distribution were compared between the groups using single-factor multiple means, and the independent sample *T* test was used between the two groups. Rank sum test was used for measurement data that did not conform to normal distribution. Chi-square test was used for counting data. Logistic multivariate analysis was used to analyze the risk factors influencing the conversion of thoracotomy to thoracotomy after thoracoscopic lung cancer resection. The difference in survival rate was analyzed by logrank test. The Kaplan-Meier test was used for univariate analysis, and COX proportional risk regression model was used for multivariate analysis. The prognostic value of lung cancer was analyzed using nomogram prediction model. *P* < 0.05 was considered as statistically considerable.

## 3. Results

### 3.1. Patients' Conversion to Thoracotomy

A total of 96 patients with non-small-cell lung cancer underwent thoracoscopic lung cancer resection in this study, including 8 patients who underwent thoracotomy, with a conversion rate of 8.33%. The reasons for conversion to thoracotomy included hemorrhage in 1 case, unclear hilar structure separation in 1 case, tumor invasion to obvious blood vessels or near hilar in 3 cases, severe adherent enlarged lymph nodes in 2 cases, and dysplasia of interlobular fissure in 1 case (Table 1).

### 3.2. Basic Patient Information

Among 96 patients with non-small-cell lung cancer, 88 patients undergoing thoracoscopic lung cancer resection were defined as the thoracoscopic group, while 8 patients undergoing conversion to thoracotomy were defined as the thoracotomy group. The basic conditions of the two groups were compared, and the results are shown in Table 2. There were no significant differences in gender ratio, mean age, and smoking history between the thoracoscopic group and the thoracotomy group (*P* > 0.05).

### 3.3. Patients' CT Manifestations

CT findings of different types of lung cancer are also different. In early central lung cancer, CT can clearly show irregular thickening of bronchial wall, lumen stenosis, lumen nodules, and other changes. In the middle and late stages, CT can clearly show intraluminal or extraluminal masses, irregular wall, and lumen stenosis. The early manifestations of peripheral lung cancer are the internal changes, marginal conditions, and peripheral signs of the tumor. CT can clearly display the edge, shape, peritumoral appearance, internal structure, and density changes of the mass in intermediate and advanced peripheral lung cancer. CT findings of diffuse lung cancer can clearly show diffuse lung cancer in both lungs, presenting as diffuse nodules in both lungs, accompanied by hilar and mediastinal lymph node metastasis.  Figure 1 shows the CT images of two NSCLC patients before and after chemotherapy. The patient had space-occupying lesions in the upper lobe of the right lung with necrosis, partial atelectasis changes, right enclosing pleural effusion, mediastinal lymph node enlargement, and effusion decreased or disappeared after chemotherapy.

### 3.4. Risk Factor Analysis of Conversion to Thoracotomy

Univariate analysis was conducted on the basic information of patients in the two groups, including age, sex ratio, smoking history, and past disease history, and the results are shown in Table 3. There was no significant difference in the proportion of patients with different gender and smoking history between the two groups (*P* > 0.05). The proportion of patients over 65 years of age, history of coronary heart disease, diabetes, and tuberculosis between the thoracotomy group and the thoracoscopic group was statistically significant (*P* < 0.05).

Single-factor analysis was conducted on the surgical methods (simple lobectomy, combined lobectomy, and segmental resection of the lung) and operative time of the two groups, and the results are shown in Table 4. The proportion of patients undergoing simple lobectomy, combined lobectomy, and segmental resection of the lung in the conversion to thoracotomy group was 2.08%, 4.17%, and 2.08%, respectively. In the thoracoscopic group, those were 34.38%, 40.63%, and 16.67%, respectively. The operation time of the conversion to thoracotomy group and the thoracoscopy group was 206.41 ± 25.27 min and 178.23 ± 20.44, respectively. Different surgical methods and operation time had statistical significance between the two groups (*P* < 0.05).

Univariate analysis was conducted on the development of interlobar fissure, pleural adhesion, postoperative chemotherapy, tumor diameter, tumor location, tumor TNM stage, and other pathological conditions in the two groups, and the results are shown in Table 5. The results showed that there were no considerable differences in postoperative chemotherapy, different tumor locations, histological morphology (squamous cell carcinoma, adenocarcinoma, and large-cell carcinoma), and histological differentiation degree (low differentiation, medium differentiation, and high differentiation) between the conversion to thoracotomy group and the thoracoscopic group (*P* > 0.05). There were statistically considerable differences between the conversion to thoracotomy group and the thoracoscopic group in the development of interlobular cleft, pleural adhesion, tumor diameter > 3.5 cm, vascular and lymph node invasion, and tumor TNM stage (*P* < 0.05).

Logistic multifactor regression analysis was performed on the seven factors with statistical significance in the above univariate analysis (age, tumor diameter, interlobular fissure development, history of tuberculosis, pleural adhesion, vascular and lymph node invasion, and TNM stage). In Table 6, patients' age ≥ 65 years, tumor diameter > 3.5 cm, interlobular fissure dysplasia, patients' history of pulmonary tuberculosis, pleural adhesion, and TNM stage IIIa were all independent influencing factors for the conversion to thoracotomy of patients with lung cancer undergoing thoracotomy.

### 3.5. Risk Factors of Thoracoscopic Resection of Lung Cancer

The results of univariate analysis of prognosis of patients undergoing thoracoscopic lung cancer resection are shown in Table 7. Tumor diameter > 3.5 cm, postoperative chemotherapy effect, surgical method, tumor TNM stage, number of chemotherapy cycles, and surgical time were all influential factors leading to poor postoperative prognosis.

Table 8, which shows the multivariate analysis of prognosis in Cox model, shows that tumor diameter > 3.5 cm, chemotherapy effectiveness, chemotherapy cycle < 4, surgery methods, and TNM stage IIIa were all independent influencing factors for prognosis of patients undergoing thoracoscopic lung cancer resection.

### 3.6. Nomogram Prediction Model

Based on the above results, tumor diameter, chemotherapy, chemotherapy cycle, and TNM stage were incorporated into the nomogram prediction model, and the results are shown in Figure 2. According to the model, tumor diameter > 3.5 cm was 50 points, chemotherapy cycle 4 was 80 points, chemotherapy effectiveness was 55 points, and TNM stage IIIa was 90 points.

Figure 3 is the calibration diagram of the prediction model. The results showed that the trend of the prediction curve of the model was basically the same as that of the actual observed curve, so the prediction ability of the model was good.

## 4. Discussion

At present, thoracoscopic surgery has become the most mainstream surgical method for lung cancer surgery. No matter if it is simple pulmonary wedge resection, pulmonary segment, and lobectomy, or even pulmonary sleeve resection involving trachea and blood vessel reconstruction, all can be completed under thoracoscopy [21]. Thoracoscopic surgery includes single-hole, two-hole, three-hole, and other incision types. Although the location, number, and size of the incision are different, the internal operation is the same, requiring radical resection and lymphatic dissection of the cancer [22]. In terms of rapid recovery of patients, thoracoscopic surgery has obvious advantages compared with traditional thoracotomy. Patients' postoperative pain is substantially reduced, postoperative recovery is fast, the incidence of complications is low, and hospital stay is greatly shortened. The clinical study of An et al. [23] showed that thoracoscopic surgery can completely achieve the same therapeutic effect as thoracotomy, complete tumor resection, and complete lymph node dissection. The 5-year postoperative survival rate was significantly better than that of traditional open surgery [24, 25]. The effect of thoracoscopic treatment depends on the doctor's technical proficiency. For example, experienced doctors can better control intraoperative bleeding to ensure patient safety. Secondly, S. Li et al. [26] showed that not all lung cancer operations are suitable for thoracoscopic surgery, and thoracoscopic surgery can be used for the treatment of patients with tumors in the lung without obvious external invasion and small lymph nodes.

However, thoracoscopic surgery has its limitations, for example, the safety of open surgery in special patients at high risk of bleeding and in special cases where bleeding occurs during surgery. In addition, it was found that due to the relatively difficult thoracoscopic operation, hemorrhage and unclear separation of hilar structure during the operation may lead to a high probability of conversion to thoracotomy. According to the results of this study, there were no statistically considerable differences between the conversion to thoracotomy group and the thoracoscopic group in chemotherapy status, different tumor locations, histological morphology (squamous cell carcinoma, adenocarcinoma, and large-cell carcinoma), and histological differentiation degree (low differentiation, medium differentiation, and high differentiation). There were statistically considerable differences between the conversion to thoracotomy group and the thoracoscopy group in the development of interlobular cleft, pleural adhesion, tumor diameter > 3.5 cm, vascular and lymph node invasion, and tumor TNM stage (*P* < 0.05). This is similar to the research results of Chen et al. [27]. The results showed that many factors, such as the patient's age, tumor diameter, development of interlobular fissure, history of pulmonary tuberculosis, pleural adhesion, vascular and lymph node invasion, and TNM stage, could be the influencing factors of patients' conversion to thoracotomy. Therefore, to prevent the occurrence of conversion to thoracotomy in patients with lung cancer during thoracotomy and improve the treatment effect, it is necessary to prevent and control several risk factors during surgery and formulate targeted treatment measures, thereby improving the clinical efficacy and prognosis of patients.

## 5. Conclusion

In this study, patients with non-small-cell lung cancer who underwent thoracoscopic lung cancer resection were selected. Univariate analysis and logistic multivariate regression were used to analyze the risk factors for conversion to thoracotomy, and nomogram prediction model was used to analyze the prognostic factors. The results showed that the age of patients ≥ 65 years old, tumor diameter > 3.5 cm, hypoplasia of interlobular fissure, history of pulmonary tuberculosis, pleural adhesion, and TNM stage IIIa were all independent risk factors for thoracoscopic resection of lung cancer to thoracotomy. Cox model and nomogram prediction model analysis showed that surgery methods, tumor diameter > 3.5 cm, chemotherapy cycle < 4, chemotherapy, and TNM stage IIIa were all independent factors influencing the prognosis of patients undergoing thoracoscopic lung cancer resection, which were of high application value in prognosis prediction of patients. The influencing factors should be prevented and controlled as much as possible during the operation of patients, so as to effectively improve the prognosis of patients.

## Figures and Tables

**Figure 1:** CT findings of lung cancer patients. (b and d) CT images of the two patients before chemotherapy, respectively. (a, c, e, and f) CT images of two patients after chemotherapy, respectively.

**Figure 2:** Nomogram prediction model for overall survival.

**Figure 3:** Calibration diagram of prediction model.

**Table 1:** Patients' conversion to thoracotomy.

Patient	Reason for conversion to thoracotomy	Cases	Proportion
Conversion to thoracotomy (*n* = 8)	Hemorrhage	1	1.04%
	Unclear hilar structure separation	1	1.04%
	Tumor invasion to obvious blood vessels or near hilar	3	3.13%
	Severe adherent enlarged lymph nodes	2	2.08%
	Dysplasia of interlobular fissure	1	1.04%
Thoracoscopic surgery (*n* = 88)		88	91.67%
Total		96	100%

**Table 2:** Basic information of patients.

Item	Category	Group		*P*
		Conversion to thoracotomy (*n* = 8)	Thoracoscopic surgery (*n* = 88)	
Gender	Male	4 (4.17%)	43 (44.79%)	0.213
	Female	4 (4.17%)	45 (46.88%)	
Mean age (years old)		58.84 ± 6.33	61.08 ± 5.21	0.325
Smoking history	Yes	4 (4.17%)	36 (37.5%)	0.698
	No	4 (4.17%)	52 (54.17%)	

**Table 3:** Single-factor analysis of conversion to thoracotomy (basic information).

Item	Category	Total	Group		*t*/*χ*^2^	*P*
			Conversion to thoracotomy (*n* = 8)	Thoracoscopy (*n* =88)		
Age	≥65	61 (63.54%)	6 (6.25%)	55 (57.29%)	8.534	0.002
	<65	35 (36.46%)	2 (2.08%)	33 (34.38%)		
Gender	Male	47 (48.96%)	4 (4.17%)	43 (44.79%)	0.897	0.356
	Female	49 (51.04%)	4 (4.17%)	45 (46.88%)		
Smoking history	Yes	40 (41.67%)	4 (4.17%)	36 (37.5%)	4.253	0.698
	No	56 (58.33%)	4 (4.17%)	52 (54.17%)		
Past medical history	Coronary heart disease	21 (21.88%)	2 (2.08%)	19 (19.79%)	25.379	<0.001
	Diabetes	23 (23.96%)	3 (3.13%)	20 (20.83%)		
	Tuberculosis	31 (32.29%)	3 (3.13%)	28 (29.17%)		

**Table 4:** Single-factor analysis of conversion to thoracotomy (operation situation).

Item	Category	Total	Group		*t*/*χ*^2^	*P*
			Conversion to thoracotomy (*n* = 8)	Thoracoscopy (*n* = 88)		
Surgical methods	Simple lobectomy	35 (36.46%)	2 (2.08%)	33 (34.38%)	4.532	0.043
	Combined lobectomy	43 (44.79%)	4 (4.17%)	39 (40.63%)		
	Segmental resection of the lung	18 (18.75%)	2 (2.08%)	16 (16.67%)		
Surgery duration (min)			206.41 ± 25.27	178.23 ± 20.44	9.512	< 0.001

**Table 5:** Single-factor analysis of conversion to thoracotomy (pathological condition).

Item	Category	Total	Group		*t*/*χ*^2^	*P*
			Conversion to thoracotomy (*n* = 8)	Thoracoscopy (*n* = 88)		
Interlobular cleft development	Fully developed	58 (60.42%)	3 (3.13%)	55 (57.29%)	21.354	<0.001
	Hypoplasia	38 (39.58)	5 (5.21%)	33 (34.38%)		
Pleural adhesions	Yes	29 (30.21%)	6 (6.25%)	23 (23.96%)	5.38	<0.001
	No	67 (69.79%)	2 (2.08%)	65 (67.71%)		
Postoperative chemotherapy	Yes	53 (55.21%)	4 (4.17%)	49 (50%)	3.577	0.534
	No	43 (44.79%)	4 (4.17%)	39 (40.63%)		
Tumor diameter	> 3.5 cm	27 (28.13%)	5 (5.21%)	22 (22.92%)	11.231	<0.001
	≤3.5 cm	69 (71.87%)	3 (3.13%)	66 (68.75%)		
Tumor location	Left lung	48 (50%)	4 (4.17%)	44 (45.83%)	9.289	0.786
	Right lung	48 (50%)	4 (4.17%)	44 (44.79%)		
Vascular and lymph node involvement	Yes	35 (36.46%)	3 (3.13%)	32 (33.33%)	4.321	0.023
	No	61 (63.54%)	5 (5.21%)	56 (58.33%)		
Histologic morphology	Squamous cell carcinomas	23 (23.96%)	1 (1.04%)	22 (22.92%)	7.391	0.112
	Adenocarcinoma	60 (62.5%)	3 (3.13%)	57 (59.38%)		
	Large-cell carcinoma	13 (13.54%)	4 (4.17%)	9 (9.38%)		
Degree of tissue differentiation	Low differentiation	24 25%)	2 (2.08%)	22 (22.92%)	6.488	0.068
	Medium differentiation	42 (43.75%)	2 (2.08%)	40 (41.67)		
	High differentiation	30 (31.25%)	4 (4.17%)	26 (27.08)		
TNM stage	I	16 (16.67%)	1 (1.04%)	15 (15.63)	6.023	0.018
	IIa	20 (20.83%)	2 (2.08%)	18 (18.75%)		
	IIb	33 (34.38%)	3 (3.13%)	30 (31.25%)		
	IIIa	27 (28.13%)	2 (2.08%)	25 (26.04%)		

**Table 6:** Logistic multifactor regression analysis of conversion to thoracotomy for thoracoscopic lung cancer resection.

Item	*B*	Standard error	Wald	df	OR	95% CI	*P*
Age ≥ 65 years old	0.696	0.433	7.348	1	3.071	0.522-5.376	< 0.05
Tumor diameter > 3.5 cm	1.238	0.421	5.042	1	4.523	0.853-6.456	< 0.05
Underdeveloped interlobular fissure	0.786	0.506	4.377	1	6.387	1.513-8.496	< 0.05
History of tuberculosis	0.913	0.384	4.256	1	5.492	1.587-9.023	< 0.05
Pleural adhesions	1.547	0.466	4.372	1	4.387	0.603-11.547	< 0.05
Vascular and lymph node involvement	2.343	0.512	5.269	1	3.211	1.322-6.763	0.052
TNM stage IIIa	1.089	0.439	4.387	1	4.023	0.465-6.029	< 0.05

**Table 7:** Univariate analysis of prognosis of patients undergoing thoracoscopic lung cancer resection.

Item	Hazard ratio (HR)	95% CI	*P*
Age	1.237	0.753-2.345	0.241
Gender	1.446	0.868-2.137	0.156
Smoking history	1.532	0.765-2.668	0.059
Tumor diameter	1.198	0.836-2.335	0.023
Postoperative chemotherapy	1.479	0.749-2.904	0.018
Tumor location	0.873	0.803-1.786	0.056
Surgery methods	0.987	0.671-2.981	0.031
TNM stage	1.399	0.903-1.995	0.017
Surgery duration	2.875	0.619-3.896	0.006
Number of chemotherapy cycles	1.056	0.946-2.017	0.028

**Table 8:** Multivariate analysis of prognosis in Cox model.

Item	Hazard ratio (HR)	95% CI	*P*
Tumor diameter > 3.5 cm	1.298	0.868-2.137	<0.05
Effective chemotherapy	2.031	0.765-2.668	<0.05
Chemotherapy cycle < 4	1.546	0.836-2.335	<0.05
Surgery methods	1.327	0.749-2.904	<0.05
Surgery duration	0.589	0.467-0.976	0.067
TNM stage IIIa	1.044	0.671-2.981	<0.05

## Data Availability

The data used to support the findings of this study are available from the corresponding author upon request.
